# HSPA5 Could Be a Prognostic Biomarker Correlated with Immune Infiltration in Breast Cancer

**DOI:** 10.1155/2022/7177192

**Published:** 2022-09-20

**Authors:** Chao Zhang, Qing Liu, Yubo Zhou, Jianfen Hua, Ruijun Su, Jun Ai

**Affiliations:** ^1^Qujing First People's Hospital, No. 1, Yuanlin Road, Qujing 655000, China; ^2^Department of Thyroid and Breast Surgery, Qujing First People's Hospital, No. 1, Yuanlin Road, Qujing 655000, China

## Abstract

**Background:**

Breast cancer (BC) is a frequent disease in females. The heat shock 70 kDa protein 5 (HSPA5) has recently been discovered to have an important function in tumor growth. However, the biological significance of HSPA5 in BC is unknown. *Material and Method*. Firstly, The Cancer Genome Atlas (TCGA) database was applied to analyze the expressions of HSPA5 in different cancer types, especially in BC. Then, the LinkedOmics database was used to screen genes coexpressed with HSPA5 in BC, presented by protein-protein interaction (PPI) and analyzed by functional enrichment analyses. Next, the Kaplan-Meier plotter was adopted to study the prognostic significance of HSPA5 and the relation between HSPA5 expression and different clinical factors in BC. Finally, the Tumor Immune Estimation Resource (TIMER) method was adopted to explore the relation between immune infiltration and HSPA5 in BC.

**Result:**

HSPA5 was highly expressed in most cancers, including BC. Genes coexpressed with HSPA5 were mainly related to endoplasmic reticulum unfolded protein response, melanosome, thyroid hormone synthesis, N-glycan biosynthesis, and so on. In the survival analysis, high HSPA5 expression indicated a poor prognosis in BC, and the expression of HSPA5 in BC was elevated after the incidence of BC, changing with different clinical factors. In the immune infiltration, HSPA5 was positively correlated with most immune cells.

**Conclusion:**

HSPA5 is an oncogene in BC progression, and it is connected with the prognosis and the immune infiltration in BC. Our findings suggest that HSPA5 could be an immunotherapy target and a prognostic biomarker in BC.

## 1. Background

Breast cancer (BC) is a frequent disease in females [1], with a certain genetic risk [2]. According to the latest global cancer statistics, the number of new BC cases reaches 2.26 million, making it the world's biggest cancer, accounting for 11.7% of all new cancer patients, and its mortality rate is about 6.6% [3]. In the early stages, 80% of patients often have breast lumps, nipple discharge, abnormal nipples, and areolas. In the middle and advanced stages, symptoms like loss of appetite, weight loss, fatigue, and anemia may appear, and some patients may also develop tumor metastases in the lung, pleura, liver, and brain [4, 5]. Due to the fact that symptoms of early BC are not obvious, most patients are already in the advanced stage at the time of diagnosis. Although more and more adjuvant treatment methods can improve the therapeutic effect of BC [6], the recurrence and metastasis of BC are still high [7]. Thus, it is urgent to find new specific BC markers to increase the clinical diagnosis rate and improve the prognosis of BC patients.

HSPA5, a member of the heat shock protein 70 (HSP70) family [8], is the master regulator of ER homeostasis [9] and participates in antiapoptosis and negative regulation of caspase [10]. Correspondingly, multiple research investigations have shown this gene is also related to the progression of some cancers. For example, Kim et al. reported that HSPA5 was related to tumor progression and could promote the survival of head and neck cancer (HNC) by maintaining lysosomal activity [11]. Teng et al. analyzed by two-dimensional gel electrophoresis and other methods that PKM2 and HSPA5 were highly expressed in high-risk endometrial cancer (EC), which could be used as potential biomarkers of EC [12]. Moreover, this gene is also actively expressed in liver cancer, glioblastoma, osteosarcoma [13], and other cancers. However, the role of HSPA5 and its carcinogenic mechanism in BC are still poorly understood, and further exploration is still needed.

In recent years, bioinformatics [14] has become an important technology for exploring molecular markers related to tumor diseases, which promotes the research progress of genomic and proteomic data. This time, we first analyze the expression and function of HSPA5 in BC through comprehensive databases, including The Cancer Genome Atlas (TCGA), LinkedOmics database, and Tumor Immune Estimation Resource (TIMER). The above analysis will provide strong evidence for exploring the mechanism of HSPA5 in the development of BC.

## 2. Material and Methods

### 2.1. TCGA Database

TCGA database contains clinical sample information of more than 20,000 patients and 33 cancers, as well as sequencing data of various omics, such as genome, transcriptome, and epigenetics, which can effectively help 1 better understand the molecular mechanism of cancer. This time, we explored the expressions of HSPA5 in different cancer types based on TCGA database.

### 2.2. The HSPA5 Coexpressed Genes in BC by LinkedOmics

LinkedOmics is an online analysis tool of TCGA database, including 3 analysis modules: LinkFinder, LinkInterpreter, and LinkCompare. Among them, LinkFinder is convenient for users to search and query information. LinkInterpreter is used to perform rich analysis of Gene Ontology (GO), biological path, network module, and other functional categories. LinkCompare uses visualization functions to compare the correlation results, and supports multigroup analysis of cancer types. Based on the above three modules, we first analyzed the genes related to HSPA5 in BC, the top 50 upregulated and downregulated genes, and the top 200 genes with significance that were displayed by heat maps and protein-protein network (PPI), respectively. Then, GO term and Kyoto Encyclopedia of Genes and Genomes (KEGG) analyses were conducted on these genes.

### 2.3. The Prognostic Analysis on HSPA5 in BC

To verify the relation between HSPA5 and the prognosis of BC patients, we analyzed the effects of different levels of HSPA5 on the probability of relapsed-free survival (RFS) and postprogression survival (PPS) by the Kaplan-Meier plotter. After that, the relation between HSPA5 and pathological parameters (pathologic stage, age, HER2 status, T stage, N stage, and M stage) in BC samples was compared in the UALCAN database to explore the therapeutic value of the gene for patients.

### 2.4. Timer Database

TIMER is an online tumor immune cell assessment tool based on TCGA, which provides researchers with the infiltration status of 6 immune cells, CD4+ T cells, B cells, CD8+ T cells, macrophages, neutrophils, and dendritic cells. Herein, based on this tool, we conducted a correlation study between 6 immune infiltrating cells and the HSPA5 gene in BC. When *P* < 0.05, the results obtained were meaningful.

## 3. Results

### 3.1. The Expression of HSPA5 in the Pan-Cancers

Based on TCGA database, we verified the expressions of the HSPA5 in different cancers. According to the results of Figures 1(a) and 1(b), the expression of the HSPA5 gene was higher in most tumors than normal groups, and in BC, it also had a higher expression in BC tumors.

### 3.2. HSPA5 Coexpressed Genes and the Functional Enrichment Analysis

Through the LinkedOmics database, we identified the positive and negative coexpressed genes associated with HSPA5 (Figure 2(a)), displayed by heat maps (Figures 2(b) and 2(c)). In the STRING database, we uploaded the coexpressed gene information related to HSPA5 and obtained a PPI network of the top 200 significant genes with 58 nodes and 411 edges (Figure 3). Then, the functional enrichment results showed that the enrichment items of these genes in biological process (BP) were response to topologically incorrect protein, response to unfolded protein, cellular response to unfolded protein (Figure 4(a)), in cell component (CC) were endoplasmic reticulum lumen, pigment granule, melanosome, oligosaccharyltransferase complex, and endoplasmic reticulum chaperone complex (Figure 4(b)), and in molecular function (MF) were disulfide oxidoreductase activity, intramolecular oxidoreductase activity, peptide disulfide oxidoreductase activity, and oligosaccharyltransferase activity (Figure 4(c)). Furthermore, the first 5 pathways for these genes enriched in KEGG were thyroid hormone synthesis, N-Glycan biosynthesis, protein export, and so on (Figure 4(d)).

### 3.3. The Prognostic Value Analysis of HSPA5 in BC

To evaluate the clinical value of HSPA5 in BC patients, we used the Kaplan-Meier mapping tool to plot the relationship between differently expressed HSPA5, RPS, and PPS in BC patients. The results demonstrated high expression of HSPA5 that indicated poor RFS (hazard ratio, HR = 1.23, log-rank *P* = 5.8*e* − 05, Figure 5(a)); on the contrary, low expression of HSPA5 promotes the probability of PPF (*HR* = 1.34, log-rank *P* = 0.013, Figure 5(b)). In addition, we made a comparative analysis between the expression of HSPA5 and clinicopathological parameters in BC. From the results in Figures 6(a)–6(f), it was found that the expression of HSPA5 in BC was all significantly higher after BC occurrence and changed with pathologic stage, age, HER2 status, T stage, N stage, and M stage. These results showed that HSPA5 could be a prognostic biomarker in BC progression.

### 3.4. Correlation Analysis between HSPA5 Gene and Tumor Immune Infiltrating Cells in BC

Based on TIMER, we analyzed the relation between the expression of HSPA5 and 6 immune infiltrating cells in BC tissues. The results in Figure 7 showed that the expression of HSPA5 was positively related to B cell (correlation = 0.159, *P* = 5.50*e* − 07), CD8+ T cell (correlation = 0.209, *P* = 4.57*e* − 11), macrophage (correlation = 0.077, *P* = 1.55*e* − 02), neutrophil (correlation = 0.212, *P* = 4.41*e* − 11), and dendritic cell (correlation = 0.158, *P* = 9.67*e* − 07). Besides, the level of HSPA5 was negatively correlated with CD4+ T cell (correlation = −0.011, *P* = 7.36*e* − 01). The finding indicates that HSPA5 might be an immunotherapeutic target in BC.

### 3.5. Network Analysis of Relation between HSPA5 and BC Clinical Factors

The Search Tool for the Retrieval of Interacting Genes (STRING) database (http://string-db.org) can critically assess and integrate protein–protein interactions (PPI), including both direct (physical) and indirect (functional) associations. To detect potential relationships among our initial candidate genes, we mapped all the genes to the STRING network and visualized the network using Cytoscape [15].

## 4. Discussion

The prevalence of BC is a significant global public health concern. Early detection of BC is the most effective way to diagnose and treat BC in time [16]. Currently, breast ultrasound is an important and reliable method for the diagnosis of BC [17]. Although blood testing is convenient for screening in asymptomatic people, there are few effective biomarkers for detecting early disease [18, 19]. Therefore, it is necessary to develop more reliable biomarkers for early diagnosis and new treatment for BC patients.

Numerous cellular activities require iron, and improper iron metabolism can potentially result in cell death [20]. A group of iron-dependent proteins, which are broken down into stages of iron absorption, use, storage, and efflux, tightly regulates the metabolism of iron. Iron metabolism genes are tightly controlled and have a coordinated feedback control over unstable iron [21]. Ferroptosis is a regulatory cell death caused by oxidative damage, but the specific molecular regulatory mechanism remains unclear [22]. Previously, HSPA5 is found to negatively regulate the ferroptosis in human pancreatic ductal adenocarcinoma, and the HSPA5-GPX4 pathway could regulate ferroptosis resistance and inhibit the anticancer activity of gemcitabine [23]. Besides, Torti and others have discussed in their article that there is a large amount of laboratory and clinical evidence that iron is closely connected with the growth and metastasis of BC [24]. BC cells increase their intracellular iron levels through various ways, such as increasing uptake and reducing outflow. In addition, breast tumor growth may potentially be aided by changes in iron metabolism in macrophages and other cells in the tumor microenvironment [25]. Therefore, we aim to explore the expression and function in BC progression.

Herein, we firstly found that the expression of HSPA5 was upregulated in most cancers, including BC. Then, we screened the HSPA5 coexpressed genes, mainly enriched in response to unfolded protein, melanosome, thyroid hormone synthesis, and N-Glycan biosynthesis. Unfolded or improperly folded proteins that accumulate in the endoplasmic reticulum's lumen trigger the unfolded protein response (UPR), a stress reaction (ER). Numerous human illnesses, including cancer, neurological and inflammatory disorders, and metabolism, are mechanistically caused by this unchecked activation. In breast tumors, some evidence suggests that chronic activation of UPR is related to treatment resistance and disease recurrence. It was reported that the role of abnormal UPR activation and overexpression of UPR components were resistant to apoptosis and drug therapy in BC [26]. Ruffolo et al. experimentally determined that breast tumors originated from melanin synthesized by breast epithelium and tumor cells. They suggested that this breast tumor should be diagnosed as a melanocyte-differentiated cancer, and melanocytes might be the basis for the formation of primary breast melanoma [27]. Recent epidemiology describes a close relationship between thyroid function and BC, which indicates that the thyroid hormone is a vital part in the development of BC. There is also clinical evidence that hypothyroidism is beneficial to the recovery of BC. Hercbergs et al. proved that L-thyroxine, T4, was an *in vitro* proliferation factor of BC cells, and in the absence of estrogen, thyroid hormone could greatly help promote the proliferation of nuclear estrogen receptor-*α*- (ER*α*-) dependent BC cells [28]. At present, people have observed changes in serum protein glycosylation in several cancers including BC [29], which indicates that serum glycans may be potential biomarkers of BC.

In the survival analysis of HSPA5 in BC, we found the high level of HSPA5 in BC patients led to poor RFS and PPS by the Kaplan-Meier plotter. To investigate whether HSPA5 could be a prognostic biomarker in BC progression, we investigated the relationship between HSPA5 and clinicopathological parameters in TCGA database. It was found the expressions of HSPA5 were differentially expressed in patients with different pathologic stage, age, HER2 status, T stage, N stage, and M stage. From these results, we can conclude that HSPA5 is highly expressed in BC tumor tissues, and the highly expressed HSPA5 has a shorter survival time than the lowly expressed HSPA5. Therefore, HSPA5 has the potential to be a new diagnostic and prognostic biomarker in BC patients.

Tumor does not simply contain tumor cells, but it consists of various cells, stromal cells, and immune cells, which constitutes the tumor microenvironment [30]. Different immune cells play different roles in tumorigenesis with their own characteristics. Currently, the promising immunotherapy refers to a therapeutic method targeting the immune function of the body for the purpose of treating diseases [31]. In this study, we observed the relation between HSPA5 and 6 immune infiltration cells. The data showed that HSPA5 was positively related with most cells, which indicated HSAP5 might be a new immunotherapeutic target in BC. In recent years, researchers found that high expression of HSPA5 is associated with antitumor cell activity, because factors such as insufficient blood supply and nutritional conditions may lead to the existence of stressful microenvironments such as hypoxia, hypoglycemia, and acidosis in tumor entities, which may lead to the overexpression of HSPA5 in tumors, which may be a defense mechanism of tumor cells under unfavorable survival conditions. As a calcium-binding protein in the endoplasmic reticulum, HSPA5 directly inhibits the activation of proapoptotic tissue components under stressful conditions and diverts folded proteins that accumulate in the endoplasmic reticulum to maintain cellular protein synthesis, thereby maintaining calcium homeostasis and the stability of the endoplasmic reticulum of tumor cells. Therefore, the high expression of HSPA5 in tumor cells has a certain protective effect on the growth of tumor cells. This has a close relationship with the biological behavior of tumor cells and can have a direct impact on the efficacy of tumor treatment. The positive expression rate of HSPA5 protein in breast cancer tissues was significantly higher than that in the group with lymph node metastasis, suggesting that those with high expression of HSPA5 protein in breast cancer tissues have a poorer prognosis. It is also suggested that HSPA5, as a new marker for breast cancer, may be a new target for breast cancer treatment, which may provide new ideas for further research on breast cancer. Our research revealed the role of HSPA5 in breast cancer through public databases and comprehensive bioinformatics analysis. However, further experiments are needed for verification.

In conclusion, the level of HSPA5 in BC tumor tissues was significantly higher, and its high expression was related to poor PFS and PPS in BC patients. In addition, HSPA5 is positively correlated with most immune infiltration cells. Based on these results, HSPA5 can be used as a potential biomarker for the diagnosis and prognosis and a new target in the immunotherapy of BC.

## Figures and Tables

**Figure 1:** The expressions of HSPA5 in the pan-cancers. (a) The expressions of HSPA5 in pan-cancers. (b) The expression of HSPA5 in BC tissues and normal tissues. ^∗∗∗^*P* < 0.001.

**Figure 2:** HSPA5 coexpressed genes and the functional enrichment analysis. (a) The HSPA5 coexpressed genes in BC. (b) The top 50 positive genes. (c) The top 50 negative genes.

**Figure 3:** PPI network of the top 200 genes with statistical significance. 58 nodes and 411 edges.

**Figure 4:** The functional enrichment analyses on the HSPA5 coexpressed genes. (a) BP. (b) CC. (c) MF. (d) KEGG pathway. The size of the dot represents the amount of gene enrichment, and different colors indicate different *P* values.

**Figure 5:** The survival curve of HSPA5 in BC. The effect of HSPA5 expression on the (a) RFS and (b) PPS, the vertical axis represents the probability, and the horizontal axis represents time.

**Figure 6:** The relation between HSPA5 and BC clinical factors. (a) Pathologic stage. (b) Age. (c) HER2 status. (d) T stage. (e) N stage. (f) M stage. ^∗∗∗^*P* < 0.001.

**Figure 7:** The relationship between HSPA5 gene and 6 immune infiltrating cells in BC.

## Data Availability

Data will be shared on request.
